RETRACTED

# Analysis of Improvement Time and Influencing Factors of Diplopia after Intermittent Exotropia in Children

**DOI:** 10.1155/2022/2611225

**Published:** 2022-03-14

**Authors:** Fei Wang, Haijing Cao, Yuan Zhang, Wenqi Wang

**Affiliations:** Department of Ophthalmology, The Affiliated Huaian No. 1 People's Hospital of Nanjing Medical University, Huaian 223300, China

## Abstract

**Objective:**

To observe and analyze the occurrence rate, improvement time, and influencing factors of diplopia after intermittent exotropia in children.

**Methods:**

A total of 135 children with intermittent exotropia treated in our hospital from February 2019 to April 2021 were recruited. A reasonable surgical plan was exerted according to the preoperative examination of the children, the children were divided into groups according to their age, degree of strabismus, visual acuity, and binocular visual function, and the postoperative diplopia occurrence rate and improvement time of diplopia in different groups were observed and compared.

**Results:**

Postoperative diplopia occurred in 74 of 135 children with intermittent exotropia, and the postoperative incidence of diplopia was 54.81%. All diplopia occurred on the first day after the operation. There were 62 cases of contradictory diplopia (83.78%) and 12 cases of fusion of powerless diplopia (16.22%). Except for 1 case of amalgamated powerless diplopia, diplopia was not significantly improved after 6 months, which seriously affected the life of the children after the second operation, and all the others were significantly improved within 90 days. The improvement time of diplopia was 3–90 days, and the average improvement time of diplopia was 13.25 ± 3.16 days. According to their age, the children were divided into the 3–6 years old group (*n* = 69), the 7–10 years old group (*n* = 47), and the 11–14 years old group (*n* = 19). Postoperative diplopia occurred in 25 cases (36.23%) in the 3–6 years old group, 34 cases (72.34%) in the 7–10 years old group, and 16 cases (84.21%) in the 11–14 years old group. There was a significant difference in the incidence of postoperative diplopia among the three groups (*P* < 0.05). There was a significant difference in the improvement time of diplopia among the three groups (*P* < 0.05). According to the degree of strabismus before the operation, the children were divided into the <50△ group (*n* = 74) and the ≥50△ group (*n* = 61). Postoperative diplopia occurred in 32 cases (43.24%) in the <50△ group and 43 cases (70.49%) in the ≥50△ group. There was a significant difference in the incidence of postoperative diplopia between the two groups (*P* < 0.05). There was a significant difference in the improvement time of diplopia among the three groups (*P* < 0.05). According to the results of the visual acuity examination, the patients were divided into the ≥0.8 (naked eye) group (*n* = 21), the ≥0.8 (ametropia) group (*n* = 32), and the <0.8 (amblyopia) group (*n* = 32). Among them, diplopia occurred in 10 cases (47.62%) in the ≥0.8 (naked eye) group, 40 cases (48.78%) in the ≥0.8 (ametropia) group, and 24 cases (75.00%) in the <0.8 (amblyopia) group. The incidence of diplopia in the <0.8 (amblyopia) group was significantly higher than that in the ≥0.8 (naked eye) group and the ≥0.8 (ametropia) group, and the difference was statistically significant (*P* < 0.05). The postoperative diplopia improvement time in the <0.8 (amblyopia) group was significantly higher than that in the ≥0.8 (naked eye) group and the ≥0.8 (ametropia) group, and the difference was statistically significant (*P* < 0.05). There was no significant difference in diplopia occurrence rate and diplopia improvement time between the ≥0.8 (naked eye) group and the ≥0.8 (ametropia) group (*P* > 0.05). According to the results of binocular visual function examination, 92 cases had a primary function, 45 cases (48.91%) had diplopia after the operation, the average recovery time of diplopia was 12.58 ± 3.16, 43 cases had no primary function, and 30 cases (69.77%) had diplopia after the operation. The average recovery time of diplopia was 13.02 ± 3.84. There was a significant difference in the incidence of diplopia between the two groups (*χ*^2^ = 5.162). There was no significant difference in the recovery time of diplopia between the two groups (*χ*^2^ = 0.570, *P* < 0.05). In 80 cases with secondary function, diplopia occurred in 36 cases (45.00%), and the average recovery time of diplopia was 10.14 ± 2.88; in 55 cases without secondary function, diplopia occurred in 39 cases (70.91%), and the average recovery time of diplopia was 14.86 ± 3.73. There was a significant difference in the incidence of diplopia between the two groups (*χ*^2^ = 8.861, *P* < 0.002). There was a significant difference in the recovery time of diplopia between the two groups (*χ*^2^ = 6.469, *P* < 0.001). In 77 cases with tertiary function, diplopia occurred in 32 cases (41.56%), and the average recovery time of diplopia was 9.61 ± 2.39; in 58 cases without tertiary function, diplopia occurred in 43 cases (74.14%), and the average recovery time of diplopia was 13.11 ± 3.05. There was a significant difference in the incidence of diplopia between the two groups (*χ*^2^ = 14.221 *P* < 0.001). There was a significant difference in the recovery time of diplopia between the two groups (*χ*^2^ = 5.355, *P* < 0.001).

RETRACTED

**Conclusions:**

The age, degree of strabismus, visual acuity, and binocular visual function of children with intermittent exotropia are significant factors affecting the occurrence rate and recovery time of diplopia after the operation. The younger the age, the smaller the degree of strabismus, the better the vision and the second or third grade of visual function, the smaller the occurrence rate of diplopia, and the shorter the recovery time of diplopia. Thus, the above influencing factors have a certain guiding significance in predicting the improvement of postoperative diplopia and the time of diplopia disappearance. The purpose of intermittent exotropia surgery in children is not only to correct eye position and improve appearance but also to establish normal retinal correspondence in order to obtain binocular monocular function. Furthermore, postoperative diplopia in children with concomitant exotropia is very common; therefore, careful examination, comprehensive analysis, and surgical plan should be designed according to the above factors. Stereoscopic vision training as early as possible after the operation is beneficial to the establishment of normal retinal correspondence and the elimination of diplopia.

## 1. Introduction

Intermittent exotropia is a type of strabismus between recessive and concomitant exotropia, which is one of the common clinical types of ophthalmopathy. Intermittent exotropia mostly occurs in children, most of them occur at the age of 4 to 15 years old, and the incidence rate is 3.42% to 3.9%, accounting for 42% of strabismus children [1–3]. Extraocular muscle atrophy, defect of fusion mechanism, and characteristics of eyeball development are the main causes of the disease. Heredity and strong light stimulation are the risk factors leading to intermittent exotropia [4, 5]. Under normal circumstances, the movement of both eyes is consistent, and you can look at the same target at the same time and image in the macula of both eyes, which can be transmitted to the visual center to form a complete and three-dimensional single object. Nevertheless, if the binocular fusion function fails to control the correct position of the visual axis, it will lead to a deviation of the visual axis. When looking at a target, one eye looks at the target, while the visual axis of the other eye is skewed outward, leading to the occurrence of strabismus. The main clinical manifestation of strabismus is exotropia, including visual fatigue, blurred vision, diplopia, nervous system abnormality, amblyopia, and limitation of eye movement [6, 7]. The frequency and angle of intermittent strabismus in children can rarely be improved by themselves and can often be transformed into constant or alternating exotropia after delaying the opportunity of treatment, resulting in the loss of binocular visual function [8]. Diplopia means that, after strabismus, the same object is projected on the noncorresponding point of the retina of both eyes; that is, it is projected on the central fovea and the peripheral retina of the strabismus eye, the object image of the fovea is in front, and the object image of the peripheral retina is in another visual direction, so one object image is perceived as two objects [9]. Diplopia can be divided into monocular and binocular diplopia. Monocular diplopia is caused by an object falling on two different parts of the retina of one eye at the same time, while binocular diplopia is triggered by a deviation in one eye, which induces one object to fall on the noncorresponding point of the retina of both eyes at the same time. That is, one image falls on the macular fovea of the fixed eye, while the other falls on the retina around the fovea of the strabismus eye [10]. A large number of clinical studies have reported that 555 of 5900 patients with strabismus surgery complained of diplopia, accounting for 9.41% [11, 12]. Scholars reported that postoperative diplopia seriously affected the quality of life of patients. Diplopia in the vast majority of patients can disappear in a short time, and persistent diplopia is rare [13]. The main risk factors of diplopia after strabismus surgery are contradictory diplopia, diplopia induced by strabismus overcorrection or undercorrection, and fusion powerless diplopia [14]. In order to observe the incidence, improvement time, and influencing factors of postoperative diplopia in children with intermittent exotropia, 135 children with intermittent exotropia who underwent intermittent exotropia surgery in our hospital from February 2019 to April 2021 were analyzed retrospectively.

RETRACTED

In this paper, we have proposed a sophisticated mechanism to observe and analyze the occurrence rate, improvement time, and influencing factors of diplopia after intermittent exotropia in children. For this purpose, a total of 135 children with intermittent exotropia treated in our hospital from February 2019 to April 2021 were recruited. A reasonable surgical plan was exerted according to the preoperative examination of the children, and the children were divided into groups according to their age, degree of strabismus, visual acuity, and binocular visual function, and the postoperative diplopia occurrence rate and improvement time of diplopia in different groups were observed and compared.

The rest of the paper is organized as follows.

In Section 2, the proposed experimental setup for the treatment of the subjected children in dedicated hospitals is presented along with proper diagnosis, selection, and rejection methods. In Section 3, various results attained through these experiments are reported along with a complete and thorough comparative analysis in terms of the numerous performance evaluation metrics, which is followed by a detailed discussion section dedicated to elaborating the performance of the proposed scheme and its various results. Finally, concluding remarks are provided.

## 2. Proposed Method: Experimental Evaluation

### 2.1. General Information

A total of 135 children with intermittent exotropia treated in our hospital from February 2019 to April 2021 were recruited. The age ranged from 3 to 14 years, with an average of 6.37 ± 2.13 years.

#### 2.1.1. Selection Criteria

1. Meet the diagnostic criteria of intermittent exotropia [15]
2. The visual acuity of poor eyes is ≥0.3, and the difference in binocular visual acuity is not more than 2 lines (international standard logarithmic visual acuity chart)
3. The equivalent spherical lens of hyperopia does not exceed +3.5 D in each eye
4. The degree of strabismus is 25 PD–50 PD
5. Preschool random point near stereoscopic examination is ≤400 arc seconds
6. There is no high regulatory aggregate/adjustment ratio
7. There is no history of intraocular surgery and history of strabismus surgery or botulinum toxin therapy
8. Do not use adjustment stitches

#### 2.1.2. Exclusion Criteria

1. Vertical strabismus, oblique muscle abnormality, dissociated vertical deviation (DVD), and AV syndrome exist at the same time and prepare for vertical transposition of horizontal muscle or oblique muscle surgery or vertical muscle surgery
2. Eye movement is restricted due to restrictive strabismus or paralytic strabismus
3. Craniofacial deformities affect the orbit
4. Suffer from ophthalmic diseases that may lead to loss of vision (except ametropia)
5. Suffer from congenital nystagmus
6. Accompanied by mental illness and cannot cooperate with the treatment of patients

### 2.2. Inspection Method

#### 2.2.1. General Inspection Items

General inspection items include gender, age of seeing a doctor, age of onset, past history and general medical history, and family history.

#### 2.2.2. Routine Ophthalmological Examination

Routine ophthalmological examination includes binocular visual acuity, binocular slit lighting biomicroscopy, excluding anterior segment diseases, and binocular direct ophthalmoscope examination, excluding fundus diseases. Among them, all patients were examined for distant vision by international standard visual acuity chart and optometry by professional optometrists in our hospital. Children aged 7 years and below were treated with atropine sulfate ophthalmic gel point for 3 days, 3 times a day. After full mydriasis and relaxation adjustment, cyclopentolate hydrochloride eye drops for mydriasis optometry were used at the age of 8 to 12 years, and compound topiramate mydriasis optometry or small pupil optometry was used at the age of more than 12 years. The binocular corrected visual acuity of all patients was more than 0.8.

RETRACTED

#### 2.2.3. Eye Position Examination

All patients had the same experienced doctor, prism plus alternating shading examination combined with corneal light mapping method, the maximum strabismus of nearsightedness (33 cm) and distance (6 m) before the operation, covering the nondominant eyes for 1 hour, looking up and down at 25 degrees of exotropia, and eye movement.

#### 2.2.4. Diplopia Examination

From the first day after the operation, except for routine examination, diplopia was examined by a red glass every day, and subjective and objective strabismus and binocular vision, including fusion range, were examined by synoptophore. Stereoscopic vision training was performed with a stereoscope on the second day after the operation, twice a day, 15 minutes per time. After discharge, they were asked to reexamine for 1 week, 2 weeks, 1 month, 2 months, 3 months, and half a year. During the reexamination, the eye position and diplopia were mainly examined, and the subjective and objective strabismus and binocular vision were examined by synoptophore. Postoperative undercorrection or overcorrection: postoperative mild undercorrection can be treated with pen tip collection training, and mild overcorrection can be observed for 3 to 6 months. If the undercorrection or overcorrection is larger (>20), it is still unable to restore the normal position through training, or there is a tendency to increase, the second surgical correction can be performed 3–6 months after the operation.

#### 2.2.5. Binocular Visual Function and Other Examinations

Check the length of the eye axis and fundus image to see if there is external rotation in the fundus. The patients were examined by synoptophore picture and near stereopsis by Titmus.

Visual function rating [16]: Level 1: simultaneous vision means that two eyes have the ability to accept the object at the same time; that is, using the synoptophore to check, both eyes can see two different and related images at the same time. Level 2: fusion refers to the ability of the brain to synthesize the same image from both eyes and form a complete impression at the perceptual level. By using the synoptophore, the eyes can see most of the same images and a small number of different images into one image. Level 3: stereopsis refers to the ability of both eyes to perceive three dimensions. Checked with a synoptophore, the eyes can synthesize two separate identical images into a stereoscopic image.

RETRACTED

### 2.3. Surgical Methods

According to the degree of strabismus seen far and near, the operation was designed according to the LMM correction of lateral rectus muscle recession, the shortening of medial rectus muscle 1 mm correction of 4–5^△^, and the correction of one eye to one segment and one recession to about 8–10^△^. Meanwhile, the age, refractive state, and binocular vision of the patients should be considered. Monocular lateral rectus recession should be performed if the strabismus is less than −25^△^, nondominant lateral rectus recession and medial rectus shortening should be performed if the strabismus degree is less than −25^△^.

Let the patient lie on his back and flush the conjunctival sac with iodine. At the same time, propofol hydrochloride is used to anesthetize the patient's surface or ketamine combined with propofol is used to anesthetize the patient. Then, the fornix conjunctival incision is selected to separate the intermuscular ligament, total internal rectus, or external rectus. At the same time, double loop suture is used. Under local anesthesia, according to the preoperative design or intraoperative reference position, the external rectus recession and internal rectus shortening are completed and finally sutured at the end of bulbar conjunctiva. After the operation, the conjunctival sac was smeared with tobramycin dexamethasone eye ointment and 0.5% levofloxacin, pranoprofen, loteprednol eye drops, or ofloxacin eye ointment was given for 7 to 15 days after the operation. All the patients were operated on by an experienced doctor.

### 2.4. Statistical Analysis

Using SPSS21.0 statistical software, before statistical analysis, the data were tested by normal distribution and variance homogeneity analysis to meet the requirements of normal distribution or approximate normal distribution, expressed as $\bar{x}\pm s$, and repeated measurement data were analyzed by repeated measures analysis of variance. *T*-test was used to compare the two groups, *n* (%) was used as an example to represent the counting data, and *χ*^2^ test was conducted to indicate that the difference was statistically significant (*P* < 0.05).

## 3. Experimental Results and Evaluations

### 3.1. Occurrence and Improvement of Postoperative Diplopia in Children with Intermittent Strabismus

Postoperative diplopia occurred in 75 of 135 children with intermittent exotropia, and the postoperative incidence of diplopia was 55.56%. Diplopia occurred on the first day after the operation. There were 62 cases of contradictory diplopia (83.78%) and 12 cases of fusion of powerless diplopia (16.22%). Except for 1 case of amalgamated powerless diplopia, diplopia was not significantly improved after 6 months, which seriously affected the life of the children after the second operation, and all the others were significantly improved within 90 days. The improvement time of diplopia ranged from 3 to 90 days, and the average improvement time of diplopia was 13.25 ± 3.16 days.

RETRACTED

### 3.2. Comparison of Postoperative Diplopia in 135 Patients with Intermittent Exotropia and Different Age Groups

According to their age, the children were divided into the 3–6 years old group (*n* = 69), the 7–10 years old group (*n* = 47), and the 11–14 years old group (*n* = 19). Postoperative diplopia occurred in 25 cases (36.23%) in the 3–6 years old group, 34 cases (72.34%) in the 7–10 years old group, and 16 cases (84.21%) in the 11–14 years old group. There was a significant difference in the incidence of postoperative diplopia among the three groups (*P* < 0.05). There was a significant difference in the improvement time of diplopia among the three groups (*P* < 0.05), as shown in Table 1.

### 3.3. Comparison of Exotropia with Different Degrees of Strabismus and Postoperative Diplopia

According to the degree of strabismus before the operation, the children were divided into the <50 group (*n* = 74) and the ≥50 group (*n* = 61). Postoperative diplopia occurred in 32 cases (43.24%) in the <50 group and 43 cases (70.49%) in the ≥50 group. There was a significant difference in the incidence of postoperative diplopia between the two groups (*P* < 0.05). There was a significant difference in the improvement time of diplopia among the three groups (*P* < 0.05), as presented in Table 2.

### 3.4. Compare of Diplopia between Different Visual Acuity and Exotropia after Surgery

According to the results of the visual acuity examination, the patients were divided into the ≥0.8 (naked eye) group (*n* = 21), the ≥0.8 (ametropia) group (*n* = 82), and the <0.8 (amblyopia) group (*n* = 32). Among them, diplopia occurred in the ≥0.8 (naked eye) group in 10 cases (47.62%). Diplopia occurred in the ≥0.8 (ametropia) group in 40 cases (48.78%). Postoperative diplopia occurred in 24 cases (75.00%) in <0.8 (amblyopia) group. The incidence of diplopia in the <0.8 (amblyopia) group was significantly higher than that in the ≥0.8 (naked eye) group and the ≥0.8 (ametropia) group, and the difference was statistically significant (*P* < 0.05). The postoperative diplopia improvement time in the <0.8 (amblyopia) group was significantly higher than that in the ≥0.8 (naked eye) group and the ≥0.8 (ametropia) group, and the difference was statistically significant (*P* < 0.05). There was no significant difference in diplopia occurrence rate and diplopia improvement time between the ≥0.8 (naked eye) group and the ≥0.8 (ametropia) group (*P* > 0.05). All data are presented in Table 3.

RETRACTED

### 3.5. Comparison of Diplopia between Different Binocular Visual Function and Exotropia after Operation

According to the results of binocular visual function examination, 92 cases had a primary function, 45 cases (48.91%) had diplopia after the operation, the average recovery time of diplopia was 12.58 ± 3.16, 43 cases had no primary function, and 30 cases (69.77%) had diplopia after the operation. The average recovery time of diplopia was 13.02 ± 3.84. There was a significant difference in the incidence of diplopia between the two groups (*χ*^2^ = 5.162). However, there was no significant difference in the recovery time of diplopia between the two groups (*χ*^2^ = 0.570, *P*=0.571). In 80 cases with secondary function, diplopia occurred in 36 cases (45.00%), and the average recovery time of diplopia was 10.14 ± 2.88; in 55 cases without secondary function, diplopia occurred in 39 cases (70.91%), and the average recovery time of diplopia was 14.86 ± 3.73. There was a significant difference in the incidence of diplopia between the two groups (*χ*^2^ = 8.861, *P* < 0.002). There was a significant difference in the recovery time of diplopia between the two groups (*χ*^2^ = 6.469, *P* < 0.001). In that, 77 cases had a tertiary function, 32 cases (41.56%) had diplopia after the operation, and the average recovery time of diplopia was 9.61 ± 2.39. In 58 cases without tertiary function, diplopia occurred in 43 cases (74.14%). The average recovery time of diplopia was 13.11 ± 3.05 d. There was a significant difference in the incidence of diplopia between the two groups (*χ*^2^ = 14.221 *P* < 0.001). There was a significant difference in the recovery time of diplopia between the two groups (*χ*^2^ = 5.355, *P* < 0.001).

## 4. Discussion

Intermittent exotropia, which is between exotropia and constant exotropia, is regarded as a medium-high exotropia, which turns into dominant exotropia after distraction, fatigue, and close reading for a long time, accounting for about 80% of exotropia [17]. Many scholars are discussing the etiology and pathogenesis of strabismus; there are probably several major factors, one of which is anatomical factors, and various developmental abnormalities of extraocular muscles, including congenital abnormalities, microstructural abnormalities, abnormalities of muscle attachment points [17]. All kinds of anomalies accumulate, aggravate, and become strabismus for a long time. Second, the function of radiation is insufficient, the fusion ability is low, the images of both eyes cannot be well integrated into one place, and the central nervous system automatically shields one of them, so the macula of both eyes is often suppressed to varying degrees. The third regulating factor is that different refractive states cause the abnormality of regulating radiation, which brings about the imbalance between eye movement and binocular vision [18–20]. Combined with these factors, the squint angle often changes within a certain range. The frequency of exotropia and the angle of exotropia in patients with intermittent exotropia rarely recover by themselves. The state of exotropia in some patients may be stable and does not develop to a certain stage, but some patients continue to develop. With the extension of time, the regulatory collection function and fusion gradually weakened, finally lost the ability of compensation, and finally developed into constant exotropia. A small degree of intermittent exotropia is often neglected and facilitates the progression of the disease, resulting in the destruction of binocular visual function and seriously promoting the development of children's visual function. However, till now, the timing and amount of surgery for intermittent exotropia have been debated by scholars, and the regression of eye position after the operation has become a consensus, but the factors and quantity that modulate the regression of eye position remain unclear [21].

RETRACTED

Scholars performed two methods and reported that the stereopsis of patients with intermittent exotropia after operation increased [22]. Li Dan et al. have surveyed different types of intermittent exotropia and indicated that surgery is helpful to the recovery of binocular regulatory set function [23]. The clinical study of binocular visual function in children with intermittent exotropia before and after operation suggests that surgical therapeutics is beneficial to the reconstruction of binocular visual function [24]. In a retrospective study on the clinical course of patients with intermittent exotropia, 73 patients with intermittent exotropia were followed up for 4 to 23 years with an average of 10 years. It was demonstrated that patients with intermittent exotropia had quantitative and qualitative improvement with the passage of time, at least in quantitative terms, and with no association with any treatment [25].

Diplopia is due to the fact that the image of the same object falls on the noncorresponding point of the retina of both eyes, which is a common complication after strabismus surgery. Diplopia in the vast majority of patients can disappear in a short period of time, and persistent diplopia is rare. The main risk factors of diplopia after strabismus surgery are contradictory diplopia, diplopia caused by strabismus overcorrection or undercorrection, and fusion powerless diplopia [26]. Exotropia mainly occurred before 12 years old, and the incidence decreased significantly after 12 years old [27]. In this study, the incidence of postoperative diplopia in children aged 3–6 years was significantly lower than that in children aged 7–14 years, and diplopia disappeared earlier. The possible reason may be that the older the child is, the more stubborn the abnormal retinal correspondence is and the deeper the inhibition is, and its perceptual and motor compensatory function is weak, so it is not easy to reestablish normal retinal correspondence. Thus, it is considered that young children have strong plasticity of binocular visual function and good compliance with binocular visual training after the operation with sufficient recovery time.

RETRACTED

In this study, the incidence of diplopia after exotropia in the ≤50^△^ group was lower than that in the >50^△^ group, but the disappearance time of diplopia symptoms in the ≤50 group was significantly earlier than that in the >50^△^ group. The incidence of postoperative diplopia with visual acuity or corrected visual acuity ≥0.8 in children with amblyopia was significantly lower than that in children with amblyopia, but the disappearance time of diplopia in the former was earlier than that in the latter. Therefore, it is suggested that the children with small strabismus and good visual acuity may have a binocular vision or two sets of retinas corresponding to normal and abnormal retinas before the operation, while the disappearance time of diplopia symptoms is related to the rapid recovery of postoperative training. Furthermore, preoperative examination and preparation should be done carefully for children with concomitant exotropia who underwent surgery in childhood. Amblyopia patients with amblyopia should be treated with amblyopia first, and ametropia had better be fully corrected. Surgery should be performed when visual acuity returns to normal or binocular visual balance, which is of significance to the stability of posterior eye position and the recovery of binocular visual function. Patients with abnormal fusion range are prone to fusion powerless diplopia after the operation, diplopia disappears for a long time, and some of them even persist. In this study, there is a case of this kind of diplopia. Moreover, there were 62 cases of contradictory diplopia and 12 cases of fused powerless diplopia after intermittent exotropia, but there was no diplopia induced by overcorrection or undercorrection of strabismus. The incidence of postoperative diplopia in children with grade 1, 2, and 3 binocular vision function was lower than that in children without them; moreover, the disappearance time of the diplopia symptoms in children with grade 2 and 3 binocular vision function was significantly earlier than that in children without them, suggesting that children with secondary and tertiary binocular visual function may have mild macular inhibition, and it is easy to restore binocular monocular function after exotropia correction, with diplopia disappearing quickly. Therefore, careful examination and analysis of binocular visual function before the operation is of certain significance to the prediction of diplopia after the operation. The elimination of postoperative diplopia is mainly through the restoration or establishment of normal retinal correspondence, the reestablishment of new abnormal retinal correspondence, continuous monocular inhibition, the sacrifice of binocular vision, and the formation of monocular vision. After the operation, we adopt the slight under correction pen tip collection training, exercise the binocular fusion function, enhance the primary, secondary, and near stereoscopic vision function of postoperative strabismus patients, and have a certain effect on the elimination of diplopia after strabismus operation. It has been reported that pressing prism can effectively improve diplopia and reconstruct visual function before strabismus correction or after overcorrection and undercorrection [28, 29]. We also revealed that the utilization of membrane pressing prism can accelerate the elimination of diplopia caused by mild overcorrection of concomitant exotropia, which is beneficial to the reconstruction of postoperative stereopsis.

RETRACTED

In conclusion, the age, degree of strabismus, visual acuity, and binocular visual function of children with intermittent exotropia are significant risk factors promoting the occurrence rate and recovery time of diplopia after the operation. The younger the age, the smaller the degree of strabismus, the better the vision, the higher the visual function, the smaller the occurrence rate of diplopia, and the shorter the recovery time of diplopia. The above influencing factors have a certain guiding significance in predicting the improvement of postoperative diplopia and the time of diplopia disappearance. The purpose of intermittent exotropia surgery in children is not only to correct eye position and improve appearance but also to establish normal retinal correspondence in order to obtain binocular monocular function. Postoperative diplopia in children with concomitant exotropia is very common. Careful examination, comprehensive analysis, and surgical plan should be designed according to the above factors. Stereoscopic vision training as early as possible after the operation is beneficial to the establishment of normal retinal correspondence and the elimination of diplopia.

## 5. Conclusion

The age, degree of strabismus, visual acuity, and binocular visual function of children with intermittent exotropia are significant factors affecting the occurrence rate and recovery time of diplopia after operation. The younger the age, the smaller the degree of strabismus, the better the vision and the second or third grade of visual function, the smaller the occurrence rate of diplopia, and the shorter the recovery time of diplopia. Thus, the above influencing factors have a certain guiding significance in predicting the improvement of postoperative diplopia and the time of diplopia disappearance. The purpose of intermittent exotropia surgery in children is not only to correct eye position and improve appearance but also to establish normal retinal correspondence in order to obtain binocular monocular function. Furthermore, postoperative diplopia in children with concomitant exotropia is very common; therefore, careful examination, comprehensive analysis, and surgical plan should be designed according to the above factors. Stereoscopic vision training as early as possible after the operation is beneficial to the establishment of normal retinal correspondence and the elimination of diplopia [29].

## Figures and Tables

**Table 1:** Comparison of postoperative diplopia results between different age groups and intermittent exotropia $\left[n\left(\%\right),\bar{x}\pm s\right]$.

Group	Number of cases	Postoperative diplopia (n, case)		Postoperative improvement time (days)	Diplopia did not disappear (N)
		Yes	None		
3–6 y group	69	25 (36.23%)	44 (63.77%)	8.89 ± 2.31	0 (0.00)
7–10 y group	47	34 (72.34%)^a^	13 (27.66%)	15.26 ± 3.45^a^	0 (0.00)
11–14 y group	19	16 (84.21%)^ab^	3 (15.79%)	19.47 ± 4.15^ab^	1 (5.26)^ab^
*χ* ^2^ */F*		22.116		92.056	6.151
*P*		<0.001		<0.001	0.046

Note: compared with the 3–6 years old group, ^*a*^*P* < 0.05; compared with the 7–10 years old group, ^*b*^*P* < 0.05.

**Table 2:** Comparison of the results of exotropia and postoperative diplopia with different degrees of strabismus $\left[n\left(\%\right),\bar{x}\pm s\right]$.

Group	Number of cases	Postoperative diplopia (n, case)		Postoperative improvement time (days)	Diplopia did not disappear (*n*, example)
		Yes	None		
<50 groups	74	32 (43.24%)	39 (56.76%)	7.17 ± 2.08	0 (0.00)
≥50 groups	61	43 (70.49%)	12 (29.51%)	14.53 ± 3.22	1 (1.64)
*χ* ^2^ */t*		10.054		16.026	1.222
*P*		0.001		<0.001	0.269

RETRACTED

**Table 3:** Comparison of diplopia results between different visual acuity and exotropia after surgery $\left[n\left(\%\right),\bar{x}\pm s\right]$.

Group	Number of cases	Postoperative diplopia (n, case)		Postoperative diplopia improvement time (days)	Diplopia did not disappear (*n*, example)
		Yes	None		
≥0.8 (naked eye) group	21	10 (47.62%)	11 (52.38%)	9.94 ± 2.54	0 (0.00)
≥0.8 (ametropia) group	82	40 (48.78%)	42 (51.22%)	10.14 ± 2.69	0 (0.00)
<0.8 (amblyopia) group	32	24 (75.00%)^ab^	8 (25.00%)	18.47 ± 3.75^ab^	1 (3.12)
*χ* ^2^/*F*		6.909		104.241	3.243
*P*		0.032		<0.001	0.197

Note: compared with the ≥0.8 (naked eye) group, ^*a*^*P* < 0.05; compared with the ≥0.8 (ametropia) group, ^*b*^*P* < 0.05.

## Data Availability

The datasets used and analyzed during the current study are available from the corresponding author upon reasonable request.
